# Elevated Serum Fibroblast Growth Factor 21 Is Relevant to Heart Failure Patients with Reduced Ejection Fraction

**DOI:** 10.1155/2022/7138776

**Published:** 2022-01-11

**Authors:** Liuzhang Fan, Lingyun Gu, Yuyu Yao, Genshan Ma

**Affiliations:** ^1^Department of Cardiology, Zhongda Hospital, Medical School of Southeast University, 87 Dingjiaqiao, Nanjing, Jiangsu 210009, China; ^2^Department of Cardiology, Fourth Affiliated Yancheng Hospital of Nantong University, Yancheng 224001, China; ^3^Department of Cardiology, Jiangyin Hospital Affiliated to Southeast University, 163 Shoushan Road, Jiangyin, Jiangsu 214400, China

## Abstract

**Objective:**

The aim of this study was to evaluate the roles of fibroblast growth factor 21 (FGF21) in heart failure patients with reduced ejection fraction and its association with Heart Failure with reduced Ejection Fraction (HFrEF).

**Methods:**

The level of FGF21 was measured by enzyme-linked immunosorbent assay (ELISA) in 199 subjects enrolled in this study, including 128 subjects with HFrEF and 71 control subjects. The mean follow-up time was 13.36 months. The left ventricular end-diastolic diameter (LVEDD) and left ventricular ejection fraction (LVEF) percentage were evaluated by the 2D echocardiography. Serum brain natriuretic peptide (BNP) was measured in the routine clinical laboratory.

**Results:**

The serum FGF21 level was evidently higher in patients with HFrEF than in the control group (228.72 ± 24.04 vs. 171.60 ± 12.98, *p* < 0.001). After 1 year of follow-up, 61 patients (47.66%) with heart failure were readmitted to the hospital, including 8 deaths (13.11%). The AUC of the receiver operating characteristic (ROC) curve for the predictive value of FGF21 for prognosis was 0.964. Kaplan-Meier analysis results showed that there were significant differences in the 1-year mortality and heart failure readmission events between the grouped subjects. A poor prognosis was correlated with the serum level of FGF21, BNP, LVEDD, and LVEF, which was confirmed by the univariate Cox analysis.

**Conclusion:**

FGF21 was independently associated with an increased risk of mortality and readmission HFrEF patients. Therefore, FGF21 has the potential to be a biomarker for the progression of HFrEF in patients.

## 1. Introduction

Heart failure (HF) is a serious clinical syndrome involving disorders of the autonomic, neuroendocrine, and immune systems. HF remains a major health threat worldwide. The global prevalence of HF is about 1-2%. Approximately 38 million people worldwide are affected by HF [1, 2]. Among patients with signs and symptoms of HF, about half of them have preserved left ventricular ejection fraction (HFpEF). Several comorbidities generally occur in both types of HF (preserved and reduced EF) [3]. In HFpEF patients, the proportion of deaths caused by cardiovascular events is higher, but the proportion of noncardiovascular deaths in HFpEF patients is higher than that in HFrEF patients. Most observational studies have shown that the mortality risk of HFpEF is similar to that of HFrEF, indicating the importance of this pathology [1–3]. Although medical treatment and patient management have evidently improved in recent decades, about 15-45% of HF patients die within one year after admission, and no more than 50% of HF patients survive for more than 5 years [1, 4]. Thus, improving risk prediction is of major importance in these patients [5, 6]. Biomarker detection is a critical approach to diagnose heart failure. This method usually detects the natriuretic peptides secreted mainly from myocardial cells in patients with heart failure due to pressure or volume overload [7, 8]. However, factors such as obesity, age, renal function, and atrial fibrillation can affect brain natriuretic peptide (BNP) levels [9]. Therefore, an objective biomarker with fewer interference factors is warranted.

Fibroblast growth factors (FGFs) are secreted proteins [10]. FGF21 is a cytokine that has the function of regulating glucose and lipid metabolism [11]. FGF21 secreted by cardiomyocytes is very important for maintaining the health of the heart. The heart is sensitive to the effects of FGF21, including systemic and local effects. This is due to the expression of *β*-Klotho in cardiomyocytes [9]. *β*-Klotho is a key coreceptor known to be specifically responsive to the effects of FGF21 [11]. Previous studies have shown that FGF21 can protect the heart from cardiomyocyte hypertrophy, ischemia, and reperfusion injury [12, 13]. The expression of FGF21 in the heart is a response to heart damage, consisting of experimental cardiac hypertrophy and myocardial infarction in rodents, as well as in failing human hearts [9–13]. In humans, circulating FGF21 levels are elevated in coronary heart disease and atherosclerosis and are related to a high risk of cardiovascular events in patients with type 2 diabetes [8–10]. In the current study, we aimed to study the association between circulating FGF21 and cardiac strength (HFrEF) for ejection studies.

## 2. Methods

### 2.1. Study Population

Study participants were 128 nonconsecutive patients with HFrEF hospitalized at the Cardiology Department of Jiangyin People's Hospital, and 71 control subjects were recruited between January 2017 and June 2018. The diagnosis of HF was based on the guidelines of the European Society of Cardiology [14]. Patients were enrolled according to the following criteria: (1) hospitalization due to cardiac decompensation, (2) New York Heart Association (NYHA) functional class III or IV at admission, and (3) left ventricular ejection fraction (LVEF) < 40%. The patient exclusion criteria were (1) thromboembolism and collagen disease; (2) severe kidney and liver diseases; (3) any malignant diseases; and (4) some inflammatory diseases, such as septicemia and septicopyemia. All HFrEF patients were treated with *β*-blockers, angiotensin-converting enzyme inhibitors, and diuretics according to the degree of ankle swelling. This study was performed based on the Declaration of the Helsinki World Medical Association. The protocols of the current study were approved by the Ethics Committee of Jiangyin People's Hospital, and informed consent forms were obtained from all participants.

### 2.2. General Information

Participants were evaluated after admission. General information of the subjects included gender, age, medication history, occupation, history of diseases, and whether there were other diseases. A standardized questionnaire was used to conduct face-to-face interviews with the patients. Systolic blood pressure (SBP), diastolic blood pressure (DBP), weight, and height are measured by trained nurses using standardized protocols. Body mass index (BMI) is calculated as weight (kg)/height^2^ (m^2^). Assessment of cardiac function capacity was done through NYHA classification.

### 2.3. Blood Sampling and Laboratory Analysis

The patient blood sample was collected after an overnight fast. Serum was obtained through centrifuging immediately at 4°C, 3000 rpm for 10 min, and stored in a refrigerator at -80°C freezer until use. The biochemical variables, such as blood urea nitrogen (BUN), serum creatinine (SCr), and serum BNP, were measured by standard methods using Roche cobas e602 and e702 in the clinical laboratory. The serum level of FGF21 was measured by enzyme-linked immunosorbent assay (ELISA) according to the R&D Systems protocol (BioVendor Group, R&D, USA).

### 2.4. Echocardiography

The 2D echocardiography was carried out by experienced operators using an ultrasound machine (Philips iE33 xMATRIX). The percentage of LVEDD and LVEF percentage were determined at the parasternal long-axis and short-axis views. All protocols were carried out following the recommendations by the American Society of Echocardiography and the European Association of Echocardiography [15].

### 2.5. Follow-Up and Study Endpoints

The time of follow-up was from the date the patients were enrolled to June 2019. All-cause mortality and readmission were chosen as the endpoints of the research. Follow-up was performed through regular outpatient interviews and monthly telephone interviews with patients or their families.

### 2.6. Statistical Analysis

Statistical analysis was performed by the SPSS 22.0 statistical package. The quantitative variables were presented as means ± standard deviations (SD) or medians (interquartile ranges). Categorical variables are presented as absolute numbers (percentages). Independent *t*-tests and chi-squared tests were performed. Pearson's correlation was employed to evaluate the correlations. Receiver operating characteristic (ROC) analysis was performed to determine better cut-off values and their corresponding sensitivity and specificity. The cut-off value was used for Kaplan-Meier analysis and Cox analysis. Cox analysis was used to analyze the independent risk factors. *p* < 0.05 was considered statistically significant.

## 3. Results

### 3.1. Patient Characteristics

In this study, 128 HFrEF patients and 71 controls were enrolled for analysis. The basic information of the participants is shown in Table 1. No differences in sex, age, BMI, BUN, or hypertension or DM history were observed among the two groups. However, all patients with HFrEF were in NYHA class III or IV. Serum levels of BNP and creatinine were significantly stronger in the patients with HFrEF than in controls. Evident differences in LVEDD and LVEF were observed between the two groups. The concentration of FGF21 was dramatically higher in the patients with HFrEF than in the control group (228.72 ± 24.04 vs. 171.60 ± 12.98, *p* < 0.001).

### 3.2. Correlation between FGF21 and Clinical Variables of HFrEF Patients

Pearson's correlation shows that there is no significant correlation between FGF21 levels and some parameters, such as gender, age, BMI, creatinine, and the history of DM or hypertension. However, FGF21 in the serum was positively correlated with BNP (*r* = 0.921, *p* < 0.001) and LVEDD (*r* = 0.814, *p* < 0.001). In addition, the serum FGF21 level was negatively correlated with LVEF (*r* = −0.853, *p* < 0.001).

### 3.3. The Prognostic Value of FGF21

61 cases of heart failure readmission (47.66%) were identified after 1 year of follow-up, including 8 cases of death (13.11%). The average follow-up time was 13.36 ± 7.54 months. To explore the independent predictors of the risk of HFrEF in patients, we performed statistical analysis. Compared with the non-endpoint event group, LVEDD, LVEF, BNP, and FGF21 in the endpoint event group displayed significant differences (Table 2). The AUC of the ROC curve for the predictive value of FGF21 for prognosis was 0.964, and the optimal cut-off value was 231.38 pg/mL, with a corresponding sensitivity of 90.2% and a specificity of 91.0% (Figure 1). Kaplan-Meier analysis and univariate Cox analysis were performed based on the performed cut-off value (Table 3, Figure 2). Kaplan-Meier analysis shows that there are significant differences in 1-year mortality and 1-year heart failure readmission events between different groups of subjects (Figure 2). The univariate Cox analysis showed that serum FGF21, BNP, creatinine, age, sex, hypertension, LVEDD, and LVEF were associated with a poor prognosis (Table 3). Therefore, FGF21 and BNP have a certain prognostic value for 1-year adverse cardiac events in patients with heart failure with a reduced ejection fraction.

## 4. Discussion

The current research represented the first study to provide evidence that the serum level of FGF21 was significantly increased in HFrEF patients. Moreover, there was a positive correlation between the circulating FGF21 and BNP levels. Our results indicated that high levels of FGF21 are independently associated with HFrEF and 1-year adverse cardiac events in HFrEF patients. Our analysis is beneficial to the comprehensive elucidation of the pathophysiological role of FGF21, which could be a potential biomarker for the presence of HFrEF and risk prediction in these patients.

Previous studies have shown that FGF21 in serum was associated with cardiovascular diseases such as diabetic cardiomyopathy, hypertensive heart disease, atrial fibrillation, coronary artery disease, and hypertension [16–22]. Moreover, FGF21 could also predict adverse cardiac events. Lakhani et al. indicated that FGF21 could dramatically predict the incidence and mortality of coronary artery disease and cardiovascular disease [23]. Previous studies have shown that the level of FGF21 in plasma is related to the diastolic dysfunction of the heart, especially in patients with heart failure with preserved ejection fraction [24]. In addition, compared with NT-pro-BNP, circulating FGF21 can better predict the presence of diastolic dysfunction and adverse cardiac events in diastolic heart failure patients within 1 year. However, previous data from patients with HFrEF are rare. Our results show that the role of FGF21 is very important, and the level of FGF21 can be upregulated during HFrEF, which can predict 1-year adverse cardiac events in HFrEF patients. The current results were in line with the evidence showing that FGF21 could protect against adverse cardiac remodeling and hypertrophy in several ways [12, 13].

Previous studies have shown that FGF21 is a marker of cardiovascular risk and can also protect the cardiovascular system [25]. First, FGF21 plays an important role in glycolipid metabolism [26]. In preclinical models of obesity and type 2 diabetes, FGF21 could improve glucose homeostasis and promote weight loss [27]. Then, FGF21 could regulate the NF-*κ*B or PI/Akt signaling pathways to alleviate the inflammatory response [9]. Besides, there is strong evidence that the AMP-activated protein kinase (AMPK)/Akt pathway is involved in cardiac protection [27, 28]. A mechanism study showed that the antiapoptotic effect induced by FGF21 in type 1 diabetes mellitus (T1DM) mice was attributed to the activation of AMPK, followed by the inactivation of phosphatase and tensin homolog (PTEN), which negatively regulates Akt signaling [9, 27, 28]. In addition, there is increasing evidence that the activation of AMPK can improve nuclear factor (erythroid-derived 2)-like 2- (Nrf2-) mediated antioxidant effect. Nrf2 is the main regulator of cell detoxification and redox state by inducing the expression of a variety of antioxidant genes. Recent studies have shown that Nrf2 agonists can prevent cardiomyopathy induced by T2DM. Further studies indicate that garlic alleviates oxidative stress in the heart by activating the Akt/Nrf2 pathway in fructose-fed diabetic rats [28].

Moreover, FGF21 plays a unique role in reducing oxidative stress in cardiomyocytes in vitro and in vivo [28]. Holm MR et al. first reported that FGF21 levels are related to cardiac cachexia. FGF21 is independently associated with IL-6, a biomarker of inflammation [29]. These functions provide conditions for FGF21 to play a cardioprotective role. Our results demonstrated that circulating FGF21 was related to BNP, LVEF, and LVEDD in heart failure subjects. Furthermore, we demonstrated the prognostic value of FGF21 among HFrEF patients. Plasma BNP levels are able to predict the incidence and mortality of cardiovascular diseases among heart failure patients and the general population [30, 31]. Besides, galectin-3 and copeptin are considered candidate biomarkers for the detection of early cardiomyopathy. At the heart level, galectin-3 expression is low, but during heart injury, it is rapidly induced [32]. The plasma galectin-3 level is considered to be a good biomarker for the prediction and prognosis of left ventricular systolic dysfunction and heart failure in diabetic patients. Galectin-3 may have therapeutic significance because its inhibitory effect can prevent proinflammatory and profibrotic mechanisms [32].

## 5. Limitations

Our results cannot fully support the substitution effect of FGF21 on BNP. However, there is a strong correlation between FGF21 and HFrEF, and our research results have a certain guiding significance for metabolic regulators in the study of HF. This study still has some limitations. First, the sample size of this study was relatively small, so we need to include a larger sample size in the future. Second, unfortunately, the level of FGF21 was measured only at a single hospital with HFrEF patients. The change of FGF21 concentration was not shown, especially during the progression of heart failure. Last, the echocardiogram is not collected at the same time. In the future, it is necessary to clearly distinguish between population studies of HF entities and experimental studies to investigate the exact pathophysiological mechanism to further clarify the different roles of FGF21 in HFrEF.

## 6. Conclusion

The FGF21 level was related to HFrEF among patients. FGF21 was independently associated with 1-year adverse events in patients with HFrEF. Therefore, FGF21 has the potential to be a biomarker for the progression of HFrEF among patients.

## Figures and Tables

**Figure 1:** ROC curve of the predictive value of FGF21 for the prognosis of patients with HFrEF.

**Figure 2:** Kaplan-Meier curve for serum FGF21 levels. The cut-off points were determined using the ROC curve.

**Table 1:** The demographic and baseline clinical characteristics of the HFrEF and control groups.

Variables	HFrEF group	Control group	*p* value
Gender (male) (*n*, %)	86 (67.19%)	51 (71.83%)	0.527
Age (years)	70.91 ± 12.378	68.00 ± 8.182	0.077
BMI (kg/m^2^)	23.303 ± 3.655	22.58 ± 1.897	0.120
Hypertension (*n*)	65	29	0.186
Diabetes mellitus (*n*)	30	12	0.365
BNP (ng/L)	2810.661 ± 1086.868	49.311 ± 21.529	≤0.001
BUN (mmol/L)	8.60 ± 3.79	7.68 ± 3.50	0.09
Creatinine (*μ*mol/L)	118.191 ± 113.209	74.732 ± 15.581	0.002
NYHA class III (%)	36 (28.13%)	—	≤0.001
NYHA class IV (%)	92 (71.87%)	—	≤0.001
LVEDD (mm)	54.59 ± 5.073	50.99 ± 3.548	≤0.001
LVEF (%)	0.321 ± 0.044	0.615 ± 0.0237	≤0.001
FGF21 (pg/mL)	228.72 ± 24.04	171.60 ± 12.98	≤0.001

HFrEF: Heart Failure with reduced Ejection Fraction; BMI: body mass index; BNP: brain natriuretic peptide; BUN: blood urea nitrogen; NYHA: New York Heart Association; LVEDD: left ventricular end-diastolic diameter; LVEF: left ventricular ejection fraction; FGF21: fibroblast growth factor 21.

**Table 2:** The clinical characteristics of the endpoint event group and non-endpoint event group.

Variables	Endpoint event group (*n* = 61)	Non-endpoint event group (*n* = 67)	*p* value
Gender (male) (*n*, %)	45 (73.77%)	41 (61.19%)	0.066
Age (years)	72.30 ± 11.62	69.66 ± 12.99	0.230
BMI (kg/m^2^)	23.04 ± 3.57	23.54 ± 3.74	0.444
Diabetes mellitus (*n*, %)	18 (29.51%)	12 (17.91%)	0.122
Hypertension (*n*, %)	36 (59.02%)	29 (43.28%)	0.075
BNP (pg/mL)	3805.59 ± 1457.07	1904.83 ± 579.05	≤0.001
Creatinine (*μ*mol/L)	139.25 ± 151.12	99.05 ± 56.00	0.046
BUN	9.58 ± 3.92	7.74 ± 3.47	0.006
LVEDD (mm)	58.51 ± 3.70	51.03 ± 3.167	≤0.001
LVEF (%)	0.28 ± 0.03	0.35 ± 0.02	≤0.001
FGF21 (pg/mL)	248.34 ± 12.16	210.85 ± 17.25	≤0.001

BMI: body mass index; BNP: brain natriuretic peptide; BUN: blood urea nitrogen; LVEDD: left ventricular end-diastolic diameter; LVEF: left ventricular ejection fraction; FGF21: fibroblast growth factor 21.

**Table 3:** Univariate Cox analysis for prognosis in patients with HFrEF.

Variables	OR value	*p* value	95% CI
Gender (male, *n*)	0.146	≤0.001	0.061-0.345
Age (years)	0.954	0.004	0.923-9.985
BMI (kg/m^2^)	0.971	0.522	0.887-1.063
Hypertension (*n*)	2.489	0.007	1.286-4.815
Diabetes mellitus (*n*)	0.602	0.154	0.300-1.210
BNP (ng/L)	1.005	≤0.001	1.003-1.006
Creatinine (*μ*mol/L)	1.003	0.002	1.001-1.005
LVEDD (mm)	0.896	0.026	0.814-0.987
LVEF (%)	≤0.001	0.005	≤0.001-≤0.001
FGF21 (pg/mL)	0.964	0.008	0.939-0.990

BMI: body mass index; BNP: brain natriuretic peptide; LVEDD: left ventricular end-diastolic diameter; LVEF: left ventricular ejection fraction; FGF21: fibroblast growth factor 21.

## Data Availability

The data used in this study can be obtained from the corresponding author upon reasonable request.
